The article "Primary and Triage Cervical Screening Diagnostic Value of Methods for the Detection of Cervical Dysplasia" was published in 2022. Journal: Biomed Res Int.

# Primary and Triage Cervical Screening Diagnostic Value of Methods for the Detection of Cervical Dysplasia

**DOI:** 10.1155/2022/1930102

**Published:** 2022-09-17

**Authors:** James Kinoti Njue, Margaret Muturi, Lucy Kamau, Raphael Lwembe

**Affiliations:** ^1^Department of Medical Laboratory Science, Kenyatta University, Kenya; ^2^Department of Animal Science, Kenyatta University, Kenya; ^3^Centre for Virus Research, Kenya Medical Research Institute (KEMRI), Kenya

## Abstract

**Background:**

Cervical cancer is a leading cause of mortality among women globally. Approaches to reduce cervical cancer incidence and mortality are “screen-and-treat,” where positive primary test only is used in the treatment and “screen, triage and treat,” where treatment is based on positive primary and triage tests with/without histological analysis.

**Objectives:**

To determine cervical screening outcomes among HIV-infected and noninfected women using VIA, Pap smear, and HPV-PCR cervical screening methods and to determine the sensitivity, specificity, PPV and NPV of VIA, Pap smear, and HPV-PCR as primary test and sequential triage based on abnormal histopathology among HIV-infected and noninfected women. *Methodology*. This was a comparative cross-sectional study where women aged 18-46 years women underwent cervical screening and colposcopy-biopsy test as a positive-confirmatory test in the Referral Hospitals of Eastern Kenya.

**Results:**

A total of 317 (HIV negative: 156/317 (49.2%) and HIV positive: 161/317 (50.8%)) women were enrolled. Of these 81/317 (25.6%), 84/317 (26.5%), 96/317 (30.2%), and 78/122 (63.9%) participants had VIA, HPV DNA-PCR, Pap smear, and cervical histology positive results, respectively; average: 27.4% (HIV positive: 21.5%; HIV negative: 5.9%). Majority of women with LSIL [17/317 (5.4%)], HSIL [22/317 (6.9%)], invasive cancer [5/317 (1.6%)], cervicitis [45/317 (14.2%], and candidiasis 47/317 (14.8%) were HIV-infected (*p* < 0.001). 78/317 (24.6%) participants had positive histology test [ASCUS: 34/317 (10.7%) CIN1:17/317 (5.3%), CIN2: 16/317 (5.0%), CIN3:6/317 (1.9%), and ICC: 5/317 (1.6%)] (*p* > 0.001). A higher primary diagnostic accuracy was established by HPV DNA-PCR (sensitivity: 95.5%; specificity: 92.6%) than Pap smear and VIA test while in triage testing, high sensitivity was obtained by HPV DNA-PCR parallel testing with VIA test (92.6%) and Pap smear test (92.7%) and VIA cotesting with Pap smear (99.9%). HIV-infected women had increased specificity and reduced sensitivity and diagnostic accuracy by both primary and triage testing approaches. *Discussion*. Abnormal cervical screening outcome was high among HIV-infected than noninfected women. HIV-infected women had significantly high cases of cervical neoplastic changes. The diagnostic value of primary tests increased upon concurrent testing with other test methods hence reducing the number of women who would have been referred for biopsy.

The article "Primary and Triage Cervical Screening Diagnostic Value of Methods for the Detection of Cervical Dysplasia" was published in 2022. Journal: Biomed Res Int.

**Conclusion:**

High sensitivity and specificity in detection of CIN+ were established among HIV-infected than HIV noninfected women by HPV DNA-PCR and Pap smear than VIA test. HPV DNA-PCR test and Pap smear are more accurate in primary and sequential triage cervical screening based on abnormal histopathology outcomes among HIV-infected than noninfected women.

## 1. Background

Cancer of the cervix is the second type of cancer among women aged 15-44 years in Kenya [1, 2]. It is primarily caused by human papillomavirus (HPV), which can be sexually transmitted and causes cervical cells neoplastic changes leading to cervical cancer [2, 3]. Wide spectra of HPV types have been established through advances in genotyping technology and classified as “high-risk” or “low-risk” HPV based on their oncogenicity [1, 4–6]. HPV deoxyribonucleic acid (DNA) replicates in the basal cells of the cervix during the initial stages of infection and integrates into the host genome. HPV cervical infection may regress and clear or progress into cervical intraepithelial neoplasia (CIN) leading to intraepithelial cellular carcinoma (ICC).

The World Health Organization (WHO) approaches to reduce cervical cancer mortality are the “screen-and-treat approach,” where the decision to treat is based on a positive primary screening test only without triage (i.e. no second screening test and no histopathological diagnosis) and the “screen, triage and treat approach,” where treatment is based on a positive primary and secondary screening test results with/without histologically confirmed diagnosis [7–10]. The WHO recommends HPV DNA detection as the primary screening test rather than visual Inspection or cytology preferably with triage in screening and treatment approaches among both the general population of women and women living with HIV [7]. Additionally, the WHO identifies research gaps and further considerations for more data on the specificity and sensitivity of cervical screening tests among women living with HIV and the impact of antiretroviral therapy (ART) on HPV-associated lesions to strengthen the screening recommendations [7].

Several visual inspections and cytologic and molecular methods are used in cervical screening to detect neoplastic cells. Visual inspection methods include less resource-intensive visual inspection with acetic acid or Lugol's iodine (VIA/VILLI) test which provides prompt results and less cytotechnology, hence excellent for low-income settings. Here, the cervix with CIN lesions is whitened following acetic acid swabbing and visualized using naked eyes, magnifying camera, colposcope, or automated digital imaging. Cytologic methods include conventional Pap smear, liquid-based cytology, and dual staining in the identification of P16 and Ki-67 cancer markers. They are more resource-intensive methods and require a laboratory for slides-staining procedures by a cytologist, and reporting by a pathologist using the Bethesda 2001 guidelines [8] takes a longer turnaround time in some cases leading to a loss of patient follow-up. Molecular methods include high-risk HPV nucleic acid amplification tests (NAAT), DNA methylation, and protein biomarkers tests for HPV antibodies and oncoprotein. They are the most resource-intensive cervical screening methods that require a specialized laboratory and highly trained personnel to carry out DNA isolation with high-cost reagents and equipment. The cervical histology method is also a high resource-intensive gold-standard confirmatory method that requires a pathologist to read slides prepared from harvested cervical samples [7–11].

The article "Primary and Triage Cervical Screening Diagnostic Value of Methods for the Detection of Cervical Dysplasia" was published in 2022. Journal: Biomed Res Int.

Literature reviews a wide range of diagnostic values in the detection of cervical dysplasia by studied population, applied methodology, and personnel. VIA screening method is associated with low specificity, while the Pap screening has reported higher specificity and sensitivity. HPV DNA-PCR method is associated with higher sensitivity, specificity, and positive predictive value (PPV) than other methods [8]. Since cervical cancer is preventable and has a longer precancerous stage, a time lasting a decade, the best and available diagnostic tools are required for early detection and management [10, 12, 13]. This precancerous stage is reduced among HIV-infected women who harbor a wide spectrum of HPV types with subsequently reduced infection clearance [5].

This study aimed to (1) determine cervical screening outcomes among HIV-infected and noninfected women using VIA, Pap smear, and HPV-PCR cervical screening methods and (2) determine the sensitivity, specificity, positive and negative predictive value, and diagnostic accuracy of VIA, Pap smear, and HPV-PCR as primary test and sequential triage based on abnormal histopathology among HIV-infected and noninfected women. These will assist in the development of effective screening strategies for early and accurate cervical abnormalities detection.

## 2. Methodology

We followed the methods described in our previous research publication [14] that focused on HPV types detected among HIV-infected and noninfected women in the same study region.

The article "Primary and Triage Cervical Screening Diagnostic Value of Methods for the Detection of Cervical Dysplasia" was published in 2022. Journal: Biomed Res Int.

This was a comparative cross-sectional study carried out in Meru, Embu, Kirinyaga, Isiolo, and Chuka Referral Hospital's Reproductive Health Clinics and HIV Voluntary Cancelling and Testing (HIV-VCT) Centers from January 2018 to December 2019. Included were consenting women aged between 18 and 47 years. Excluded were menstruating, pregnant, and mentally incompetent women and those with an eroded cervix or a history of ablative procedures or medical treatment for cervical disease in the last six months [15].

### 2.1. Human Immunodeficiency Virus Determination

HIV serostatus was determined as per the national algorithm. Alere Determine®HIV-1/2 test (Abbott Laboratories, Abbott Park, IL) was used as a baseline screening test, First Response® HIV 1-2-0 card test (Premier Medical Corporation, Nani Daman, India) as a confirmatory test, while Uni-Gold™ Recombigen® HIV-1/2 (Trinity Biotech Jamestown, New York, US) was used as a tie-breaker test [13, 15].

### 2.2. Collection and Storage of Cervical Exfoliated Cell Samples

A disposable speculum was prewarmed in sterile warm distilled water and then lubricated before use. It was then used to examine the external genitalia and locate the cervical opening (OS) while the participant lays in a lithotomic position [7, 13, 16]. The mucus plug in OS was removed and wiped to ensure sufficient cells were collected. A cervical broom (Dacron cervical broom; Digene Corporation, Silver Spring, Maryland STM™) was softly rotated 360 degrees five times to exfoliate cells from the region of the transformation zone, squamocolumnar junction, and endocervical canal. Exfoliated cells were spread evenly and fixed immediately on a clean glass slide. The broom bristles were then dipped into Aqueous Minimum Essential Media (MEM), and the broom handle snapped so that it remained in the tightly closed vial stored at 1-4° C as described by the WHO guidelines [8, 17].

### 2.3. Visual Inspection by Acetic Acid Test

The cervix was smeared with a 3-5% acetic acid solution and observed under sufficient light after 30-60s for acetowhitening around the cervical transformation zone. The test was reported as positive if acetowhitening occurred and negative if there was no acetowhitening [18, 19].

### 2.4. Cytology

A standardized protocol for Pap smear staining and examination was followed to detect cellular charges to the nuclei and cytoplasm following HPV infection. Cytopathologists supervised by a pathologist at Embu and Meru Hospitals were required to fill a pathology synoptic reporting form using the Bethesda 2001 guidelines for reporting Pap smear slides using a binocular microscope. Slides were later transferred to Kenya Medical Research Institute (KEMRI) for examination by a pathologist for results confirmation. Pap smear results were classified as normal or abnormal (ASCUS, CIN1, CIN2, CIN3, or ICC) [8].

The article "Primary and Triage Cervical Screening Diagnostic Value of Methods for the Detection of Cervical Dysplasia" was published in 2022. Journal: Biomed Res Int.

### 2.5. Polymerase Chain Reaction Test

All samples underwent HPV DNA nested PCR by the following procedure:

#### 2.5.1. DNA Extraction

Samples were subjected to the kit protocol to obtain DNA extracts by magnetic bead technique using a 96-well format HighPrep™ Viral-DNA/RNA, MagBio Genomics, Inc. USA/Canada Lysis kit and eluate stored at -20° C [7, 20, 21].

#### 2.5.2. HPV Detection

This was achieved by amplifying an L1 portion of the HPV genome that is relatively conserved through L1 consensus nested PCR in the ABI-thermocycler Model 9600, Applied Biosystems® using HPV consensus primary primers PGMY09 (GCACAGGGACATAACAATGG) and PGMY11 (CGTCCCAAAGGAAACTGATC) [15] that target the 450 bp region in the L1 ORF. Additional primer sets targeting the same region of L1, MGP5+(ACGTTGGATGTTTGTTACTGTGGTGGATACTAC), and MGP6+(ACGTTGGATGGAAAAATAAACTGTAAATCATATTCCT) were used to produce shorter amplicon of ~160 bp in nested PCR [10, 15]. Positive control of CIN2+ and negative control of distilled water were incorporated in all primer cycles [21–23]. Working stock of 5*μ*MPGMY09 primer (50 *μ*L PGMY09 100 *μ*M primer) and 5*μ*MPGMY115*μ*M (50 *μ*L PGMY11 100 *μ*M primer) were added to 350 *μ*L and 750 *μ*L molecular biology-grade water, respectively, and each filled to 1 mL total volume. They were later distributed each 5 *μ*M working stock in 45–90 *μ*L aliquots and stored at -20°C [8, 9].

In the primary PCR, 5 *μ*L of the extracted DNA was amplified in a reaction mix containing 1× PCR buffer 2.0 mM MgCl2, 500 nM forward primer MY09, 500 nM reverse primer MY11, and 100 *μ*M of each dNTPs and 0.13 units of *Taq* polymerase enzyme. In the nested PCR, 5 *μ*L of the primary PCR product, 2.0 mM MgCl2, 500 nM of GP5+, 500 nM of GP6+, and 400 *μ*M of dNTPs and 0.13 units of *Taq* polymerase enzyme were used. The cycling conditions were as follows: in primary PCR, initial denaturation at 95°C (4 minutes), the reaction was cycled 30 times at 95°C (20 sec), 56°C (40 sec), and 72°C (2 minutes) and then final extension at 72°C (7minutes), and in nested PCR, initial denaturation at 95°C (4minutes), cycling at 95°C (20 seconds), annealing at 60°C (40seconds), extension at 72°C (7seconds), and then final extension at 72°C (7minutes) [8, 16].

#### 2.5.3. Gel Electrophoresis and Visualization

The positive PCR products were purified using the QIAquick DNA purification kit™ Qiagen, Germany [21, 22]. 5 *μ*l aliquot of the product was mixed with 1 *μ*l of 6× loading dye and loaded onto a 2% agarose with 2 *μ*l ethidium bromide gel alongside a 100 bp ladder for gel electrophoresis and ultraviolet visualization using 4% agarose-Tris-Borate-EDTA 10×. The presence of the expected 160 bp amplicon was considered positive for HPV DNA PCR [7].

The article "Primary and Triage Cervical Screening Diagnostic Value of Methods for the Detection of Cervical Dysplasia" was published in 2022. Journal: Biomed Res Int.

### 2.6. Histology

All positive VIA, Pap smear, and HPV DNA-PCR participants underwent colposcopy and biopsy (as a Gold Standard method) [8]. If the result of the colposcopy was normal and satisfactory, it was considered negative, and in the case of abnormal or unsatisfactory colposcopy for the person, biopsy or endocervical curettage (ECC) was performed, and a sample was sent to the Pathology Department-KEMRI. If the report of pathology indicates an ASCUS, CIN lesion, or higher, it was considered a positive result. All biopsy samples alongside cytology reports were reviewed by a pathologist [21–23].

### 2.7. Statistical Analysis

Study results were analyzed using SPSS V16 software. Specificity, sensitivity, positive predictive value (PPV), negative predictive value (NPV), and diagnostic accuracy are presented as percentages in primary and sequential triage by using confirmed abnormal histological analysis as gold standard. Cervical screening results by VIA, Pap smear and HPV-PCR cervical screening methods are presented as numbers and percentages. The level of significance was lower than 0.05.

### 2.8. Ethical Consideration

This study was approved by the KEMRI Scientific and Ethical Review Unit (approval number: KEMRI/- SERU/CVR/004/3342). Participants were required to sign a consent here all steps and procedures for HIV and cervical exfoliated cell sample collection; analysis and collection of their results were explained.

## 3. Results

### 3.1.  Table 1: Social Demographic Characteristics and HIV Serostatus of Participants

A total of 156/317 HIV-negative and 161/317 HIV-positive women were recruited. Most participants recruited into the study were residents from Embu County [85 (26.8%)], aged ≤35 years [219 (69.1%)], were educated up to secondary school level [135 (42.6%)] and married [226 (71.3%)], and those with low-income status earning less than $1.90 per day [208 (65.6%)]. Age was significantly associated (*p* = 0.016) with HIV status: more women aged below 35years had a higher HIV infection rate than those aged over 35 years (Table 1).

### 3.2. Figure 1: Cervical Screening Results by HIV Status of Participants

Pap smear test produced most abnormal cytology results (96/317 (30.2%)) than other VIA tests (81/317 (25.6%)) and HPV-DNA-PCR (84/317(26.5%)) which were confirmed by histology (78/122 (63.9%) cervical screening outcome. A significantly higher HPV infection, positive VIA test, abnormal cytology, and histology rate were established among HIV-infected than noninfected women (*p* < 0.001) (Figure 1).

The article "Primary and Triage Cervical Screening Diagnostic Value of Methods for the Detection of Cervical Dysplasia" was published in 2022. Journal: Biomed Res Int.

### 3.3. Figure 2: Association between Pap Smear Cytological Analysis and Human Immunodeficiency Virus (HIV) Status

There was a significant association between abnormal cytology outcomes and HIV infection where the majority of women with LSIL [17/317 (5.4%)], HSIL [22/317 (6.9%)], invasive cancer [5/317 (1.6%)], cervicitis [45/317 (14.2%], and candidiasis 47/317 (14.8%) were HIV-infected (*p* < 0.001) (Figure 2).

### 3.4.  Table 2: Comparison of Cervical Screening Methods Results with Histology Outcome

Overall, 78/317 (24.6%) participants had positive histology tests which were significantly associated with other cervical diagnostic methods test outcomes. Several CIN1+ cases were reported as normal by VIA (CIN1: 1/78), HPV DNA-PCR (CIN2, 3 and ICC: 1/78), and Pap smear test (CIN1: 2/78, CIN3: 3/78, and CIN3: 1/78). However, the number of these cases was reduced upon triage testing by VIA-Pap smear test (CIN1:1/78) and Pap smear-HPV DNA-PCR (CIN1:2/78) (Table 2).

### 3.5.  Table 3: Sensitivity, Specificity, Diagnostic Accuracy, and Positive and Negative Predictive Value of Cervical Screening Methods by Histology Outcome

HPV DNA-PCR had the highest sensitivity (61.9%), positive predictive value (61.9%), and diagnostic accuracy (81.7%), while Pap smear had the highest specificity value (87.0) in the primary testing approach. HPV DNA-PCR cotesting with Pap smear showed the highest specificity (95.4%), diagnostic accuracy (94.3%), and the highest negative predictive value when cotested with the VIA test (99.9%) in triage testing. All screening methods results were significantly associated with histological confirmation (*p* < 0.001) (Table 3).

There was reduced sensitivity and increased specificity among HIV-infected than noninfected women in the primary and triage cervical screening approach. There was no difference in NPV by primary or triage screening approach but the diagnostic accuracy increased by HIV-negativity status in all approaches (Table 4).

### 3.6. Figure 3

Agaraose gel electrophoresis (2%) of PCR product. Lane T1: Size marker (500kb ladder); Lane T2: negative control; Lane T3: positive control; Lane T4 and T5: negative for HPV PCR product; Lane T6-T8: positive for HPV PCR product.

## 4. Discussion

This study used cervical histology outcomes to evaluate the diagnostic value of VIA, Pap smear, and HPV-PCR cervical screening methods in “screen-and-treat” and “screen, triage and treat” approaches among HIV-infected and noninfected women. This allows the findings to be pursued in a range of low- and middle-income settings with limited public health resources for early detection and treatment of cervical neoplasia.

The article "Primary and Triage Cervical Screening Diagnostic Value of Methods for the Detection of Cervical Dysplasia" was published in 2022. Journal: Biomed Res Int.

On average, HIV-infected women had significantly high abnormal cervical screening outcomes by all methods and HIV status (average: 27.4% (HIV infected: 21.5%; HIV noninfected: 5.9%)). Pap smear test reported high abnormal cervical screening outcomes (30.2%) than other methods. A high HIV infection rate was also established by Pap smear outcome of *Candida* spp. and bacterial infection that is associated with cervical basal layer disruption allowing HPV and HIV entry [24, 25]. HIV infection has been detailed to favor HPV acquisition and persistence [4, 23]. This could be the reason for the higher HPV infection rate and varying degrees of cervical inflammation from mild to severe among HIV-infected women in this study and others [3, 23, 24]. Abnormal histology results are 63.1% (78/122); ASCUS and higher lesions (CIN1, CIN2, CIN3, and SCC and ICC) showed significant association (*p* < 0.001) with VIA test (25.6%), Pap smear (30.2%), and HPV DNA-PCR (26.5%) results. There is growing evidence regarding the impact of ART among HIV-infected women on HPV-associated lesions [8] which calls for further studies.

The diagnostic value of primary test with VIA (true positive (TP): 16.4%; true negative (TN): 61.2%; false negative (FN): 14.2%; and false positive (FP): 8.2%) significantly reduced upon concurrently testing with Pap smear (TP: 14.5%; TN: 57.7%; FN: 6.3%; and FP: 14.5%) and HPV DNA-PCR. False-positive results that are incorrect outcomes of lesion-free women as CIN+ and FN results where CIN+ cases are not detected are a common occurrence in cervical screening [24]. Papillomavirus DNA-PCR primary testing produced negative results of ASCUS (7.3%) and in each category of CIN+ (0.3%) positive samples. However, CIN1, CIN2, CIN3, and ICC had 3.5%, 5.4%, 4.7% 1.6%, and 1.3% HPV true-positive tests, respectively. These values decreased upon triage test of HPV DNA-PCR with VIA (2.2%, 4.4%, 3.8%, and 1.6% for ASCUS, CIN1, CIN2, and CIN3, respectively). Failure to detect HPV in CIN+ samples occur in HPV false-negative case as seen in this study or when the cervical abnormality is misclassified and when the cervical abnormality is HPV-independent [24]. When Pap smear abnormal samples were subjected to HPV DNA-PCR test, the number of TP (15.8%) and TN (65.6%) reduced to 14.8% and 58.4%, respectively. Literature review triage testing produces minimal FP and FN than primary testing alone as established in this study. Therefore, primary results are applied in the “screen-and-treat approach”; greater populace benefits but the approach may lead to unnecessary treatment of negative cases or ignoring positive ones hence allowing widow neoplastic changes to occur leading to cervical cancer as well as delay early detection [24–27].

The article "Primary and Triage Cervical Screening Diagnostic Value of Methods for the Detection of Cervical Dysplasia" was published in 2022. Journal: Biomed Res Int.

In cervical screening, specificity, PPV, and diagnostic accuracy of a screening method are reflexes of FP outcome which can be a result of abnormal cervical cytology cases that spontaneously regress without progressing to cervical neoplasia upon biopsy [24]. In this study, the VIA test had the highest false-positive result [52/317 (16.4%)] than Pap smear [32 (10.1%)] and HPV DNA-PCR [31 (0.9%)] resulting in low sensitivity, specificity, and PPV (probability that a positive test is a true positive) and NPV (negative test is a true negative) as reported in other studies [24, 25]. VIA sensitivity, specificity, NPV, and diagnostic accuracy were notably high among HIV-infected than noninfected women.

Test sensitivity and negative predictive value increased when (1) a triage testing approach was applied instead of primary testing, (2) when HPV DNA-PCR was part of any triage, and (3) when applied for the detection of CIN+ without ASCUS. Sensitivity in the detection of ASCUS with CIN+ by VIA (53.6%), HPV-DNA-PCR (61.9%), and Pap cytology (61.7%) increased to 92% (VIA–Pap), 84.3% (HPV DNA-PCR–VIA), and 90.4% (Pap–HPV DNA-PCR) hence reducing the number of women who would have been referred for colposcopy in a resource-constrained setting. Specificity and PPV were high in (1) primary and triage cervical screening approach when confirmed with CIN+ without ASCUS and (2) among HIV-infected than noninfected women. The reason could be that there was a high number of true-positive cases obtained when CIN+ samples were applied in confirmation unlike when ASCUS and CIN+ were combined. Latent and initial stages of HPV infection often have a low incidence of cervical neoplasia and a higher chance of false-negativity as the viral load is too low to be detected using HPV-PCR [28].

HIV-infected women showed reduced FP and FN and increased TN results than HIV noninfected in both primary and triage tests and hence increased specificity and sensitivity by all cervical screening methods. The reason could be HPV regression upon acquisition among HIV-infected women is low meaning that most infections will progress into cervical lesions and test positive by all cervical screening methods decreasing the number of false positives and increasing true positives.

This study, therefore, agrees with one of the seven prioritized WHO algorithms for HPV DNA detection in a screen, triage and treat approach [7]. The use of this algorithm in this study significantly reduced the high number of HIV noninfected than HIV-infected women who would have undergone treatment if the primary screening approach alone was used.

The article "Primary and Triage Cervical Screening Diagnostic Value of Methods for the Detection of Cervical Dysplasia" was published in 2022. Journal: Biomed Res Int.

The strength of this study was performing cervical screening on all participants using a primary and triage screening approach that led to accurate reporting and appropriate referral based on CIN+ histological outcomes, especially among HIV-infected women as recommended by WHO.

## 5. Conclusion

The clinical relevance of cervical screening is highly dependent on the sensitivity, specificity, positive and negative predictive, and diagnostic values of screening modalities. Pap smear tests produced more positive outcomes by HIV serostatus than other cervical screening methods. High sensitivity and specificity in detection of CIN+ were established among HIV-infected than HIV noninfected women by HPV DNA-PCR and Pap smear than VIA test. HPV DNA-PCR and Pap smear tests were also more accurate in primary and sequential triage cervical screening based on abnormal histopathology outcomes among HIV-infected than noninfected women. A high diagnostic value was obtained by all cervical screening methods when CIN+ histopathology outcome was used as a reference than CIN+ with ASCUS.

## 6. Recommendation

Values obtained and accuracy of results interpretation may differ with other studied populations and hence the need for expanded studies in other regions. More longitudinal data are needed on the effectiveness and cost-effectiveness of different cervical cancer screening strategies in cervical cancer reduction, especially among HIV-infected women.

## Figures and Tables

**Figure 1:** Cervical screening results of HIV-infected and noninfected participants by visual inspection with acetic acid, HPV DAN-PCR, Pap smear, and histology. The graph shows the cervical screening outcome by human immunodeficiency virus status (average: 27.4% (HIV positive: 21.5%; HIV negative: 5.9%) of participants (*N* = 317) by visual inspection with a 3-5% acetic acid test (VIA test), Human Papillomavirus Deoxyribonucleic Polymerase Chain Reaction (HPV DNA-PCR), and Pap smear test. All participants with positive or abnormal results (*n* = 122) were referred for a colposcopy examination followed by a cervical histologic confirmatory test.

**Figure 2:** Pap smear cytological results of HIV-infected and noninfected women. The graph shows the cytology Pap smear outcome of all HIV-infected and noninfected participants presented in two categories: cytological analysis (*n* = 317) and infections and cervical abnormalities detected (*n* = 317). In the first category, 221/317 participants had normal cytology, while others (96/317) had abnormal cytology reported as atypical squamous cells of undetermined significance (ASCUS) and cannot exclude HSIL (ASC-H), low-grade Intraepithelial Lesions (LSIL), high-grade intraepithelial lesions (HSIL), and invasive cervical cancer (ICC). In the other category, cervical infections (bacterial vaginitis, candidiasis caused by Candida albicans, and trachomatis caused by Chlamydia trachomatis) are shown alongside unknown cervical inflammation.

The article "Primary and Triage Cervical Screening Diagnostic Value of Methods for the Detection of Cervical Dysplasia" was published in 2022. Journal: Biomed Res Int.

**Figure 3:** Gel electrophoresis image of secondary PCR product using a 5000 bp Ladder.

**Table 1:** Social demographic factors and HIV serostatus of participants.

Characteristics	Category	HIV serostatus [*N* (%)]		Total (*N* = 317)	*p* value
		HIV negative	HIV positive		
Residence	Embu	41 (12.9)	44 (13.9)	85 (26.8)	0.359
	Isiolo	38 (12.0)	26 (8.2)	64 (20.2)	
	Kirinyaga	23 (7.3)	33 (10.4)	56 (17.7)	
	Meru	40 (12.6)	41 (12.9)	81 (25.6)	
	T. Nithi	14 (4.4)	17 (5.4)	31 (9.8)	

Age	≤35 years	69 (21.8)	93 (29.3)	162 (51.1)	0.016∗∗
	>35 years	87 (27.4)	68 (21.5)	155 (48.9)	

Education level	Primary	43 (13.6)	53 (16.7)	96 (30.3)	0.216
	Secondary	70 (22.1)	65 (20.5)	135 (42.6)	
	College	37 (11.7)	30 (9.5)	67 (21.1)	
	University	6 (1.9)	13 (4.1)	19 (6)	

Marital status	Married	117 (36.9)	109 (34.4)	226 (71.3)	0.416
	Separated	14 (4.4)	18 (5.7)	32 (10.1)	
	Single	19 (6)	22 (6.9)	41 (12.9)	
	Divorced	6 (1.8)	12 (3.7)	18 (5.7)	

Income status§	Low	106 (33.4)	102 (32.2)	208 (65.6)	0.495
	Middle	45 (14.5)	50 (15.8)	95 (30.0)	
	High	5 (1.6)	9 (2.8)	14 (4.4)	

Total		156 (49.2)	161 (50.8)	317 (100)	

T. Nithi: Tharaka-Nithi County, §Income: low (1.90), middle (1.9-5.5), and high (>5.50) US$ PPP/day), ∗∗: the probability at the 0.05.  Table 1 shows the total number of HIV-infected and noninfected women participants. It does not represent HIV prevalence in the region since most HIV-positive participants were recruited purposively from HIV Voluntary and Testing Centers (VCT) and Reproductive Health Clinics. This enabled in recruiting of a target population of HIV-infected participants.

**Table 2:** Cervical screening methods result from histology outcome of ASCUS and CIN+.

Cervical screening methods and results	Result category	Categories of histological analysis (*N* = 78)					Positive (ASCUS, CIN+)	Negative	Total	*p* value
		ASCUS	CIN1	CIN2	CIN3	ICC				
*Primary screening approach*										
Positive VIA test										
Normal	FP	24 (7.6)	2 (0.6)				26 (8.2)	194 (61.2)	220 (69.4)	0.001∗
Abnormal	TP	10 (3.2)	15 (4.7)	16 (5.0)	6 (1.9)	5 (1.6)	52 (16.4)	45 (14.2)	97 (30.6)	
Positive HPV DNA-PCR										
Negative	FP	23 (7.3)		1 (0.3)	1 (0.3)	1 (0.3)	26 (8.2)	207 (65.3)	233 (73.5)	0.001∗
Positive	TP	11 (3.5)	17 (5.4)	15 (4.7)	5 (1.6)	4 (1.3)	52 (16.4)	32 (10.1)	84 (26.5)	
Positive Pap smear test										
Normal	FP	22 (6.9)	2 (0.6)	3 (0.9)	1 (0.3)		28 (8.8)	208 (65.6)	236 (74.4)	0.001∗
Abnormal	TP	12 (3.8)	15 (4.7)	13 (4.1)	5 (1.6)	5 (1.6)	50 (15.8)	31 (9.8)	81 (25.6)	
*Triage screening approach with positive primary test*										
Positive VIA test										
Pap smear										
Normal	FP	3 (0.9)	1 (0.3)				4 (1.3)	11 (3.5)	3 (0.9)	0.001∗
Abnormal	TP	9 (2.8)	14 (4.4)	13 (4.1)	5 (1.6)	5 (1.6)	46 (14.5)	20 (6.3)	46 (14.5)	
Total		12 (3.8)	15 (4.7)	13 (4.1)	5 (1.6)	5 (1.6)	50(15.8)	31 (9.8)	50 (15.8)	
Positive HPV DNA-PCR										
VIA test										
Normal	FP	2 (0.6)	2 (0.6)	3 (0.9)	1 (0.3)		8 (2.5)	13 (4.1)	21 (6.6)	0.001∗
Positive	TP	7 (2.2)	14 (4.4)	12 (3.8)	5 (1.6)	5 (1.6)	43 (13.6)	20 (6.3)	63 (19.9)	
Total		9 (2.8)	16 (5.0)	15 (4.7)	6 (1.9)	5 (1.6)	51 (16.1)	33 (10.4)	84 (26.5)	
Abnormal Pap smear										
DNA-PCR										
Negative	FP	3 (0.9)	1 (0.3)	1 (0.3)			5 (1.6)	21 (6.6)	3 (0.9)	0.001∗
Positive	TP	7 (2.2)	14 (4.4)	15 (4.7)	6 (1.9)	5 (1.6)	47 (14.8)	24 (7.6)	47 (14.8)	
Total		10 (3.2)	15 (4.7)	16 (5.0)	6 (1.9)	5 (1.6)	52 (16.4)	45 (14.2)	52 (16.4)	
Total		34 (10.7)	17 (5.3)	16 (5.0)	6 (1.9)	5 (1.6)	78 (24.6)	239 (75.4)	317 (100.0)	0.001∗

VIA test: visual inspection with acetic acid test; HPV DNA-PCR: human papillomavirus deoxyribonucleic polymerase chain reaction; Abnormal histology: ASCUS: atypical squamous cells of unknown significant; CIN2+: cervical intraepithelial neoplasia; and ICC: intraepithelial cervical carcinoma; ∗: the probability at the 0.001 level; FP: false positive; TP: true positive.  Table 2 shows the Primary cervical screening approach where results obtained by VIA, HPV-PCR, and Pap smear are categorized as positive, negative, normal, or abnormal by histology reports of ASCUS and CIN+ including ICC. In the triage screening approach, positive primary test results are combined with triage test results and categorized by histology report. Total positive results of ACSUS, CIN1, 2,3, and ICC are also shown alongside negative samples and total (*N* = 317).

The article "Primary and Triage Cervical Screening Diagnostic Value of Methods for the Detection of Cervical Dysplasia" was published in 2022. Journal: Biomed Res Int.

**Table 3:** Diagnostic value of cervical screening approaches in comparison with Histology results.

Cervical screening methods and approaches	Abnormal histology (%)										*p* value
	ASCUS and CIN +					CIN+					
	Sensitivity	Specificity	PPV	NPV	D/A	Sensitivity	Specificity	PPV	NPV	D/A	
*The primary cervical screening approach*											
VIA test	53.6	81.2	53.6	81.2	77.6	95.5	79.9	43.3	99.1	82.0	0.001
HPV DNA-PCR	61.9	86.6	61.9	86.6	81.7	93.2	84.2	48.8	98.7	85.5	0.001
Pap smear	61.7	87.0	61.7	87.0	81.4	86.4	84.2	46.9	97.5	84.5	0.001
*Triage cervical screening approach*											
VIA and Pap smear	92.0	64.8	69.7	67.6	90.0	83.3	72.0	16.1	98.5	72.7	0.001
HPV-PCR and VIA test	84.3	94.7	68.3	90.7	84.2	99.9	93.1	11.1	99.9	93.1	0.001
Pap and HPV DNA-PCR	90.4	95.4	66.2	89.4	94.3	99.0	95.0	15.4	99.9	95.0	0.001

VIA test: visual inspection with acetic acid test; HPV DNA-PCR: human papillomavirus deoxyribonucleic polymerase chain reaction; Abnormal histology: ASCUS: atypical squamous cells of unknown significant; CIN2+: cervical intraepithelial neoplasia (CIN2+); and ICC: intraepithelial cervical carcinoma; sensitivity = TP/(TP + FN); specificity = TN/(TN + FP); positive predictive value (PPV) = TP/(TP + FP); negative predictive value (PPV) NPV = TN/(FN + TN); diagnostic accuracy = TP + TN/TP + TN + FP + FN, where TP = true positive; FP = false positive; TN = true negative; FP = false positive and *p* value: probability at the 0.001 level.

**Table 4:** Diagnostic value of cervical screening methods and approaches in comparison with histology results by HIV serostatus.

Cervical screening approach and methods	HIV status	Diagnostic values of cervical screening methods					*p* value
		Sensitivity	Specificity	PPV	NPV	D. accuracy	
The primary cervical screening approach							
VIA	Negative	75.0	91.2	31.6	98.5	92.5	0.001
	Positive	88.9	76.0	51.6	96.0	91.0	
Pap smear	Negative	87.5	91.2	35.0	99.3	93.5	0.001
	Positive	97.2	66.4	45.5	98.8	86.6	
HPV DNA-PCR	Negative	87.5	94.6	46.7	99.3	96.7	0.001
	Positive	97.2	72.8	50.7	98.9	91.5	

Triage screening approach							
VIA test–Pap smear	Negative	75.0	95.3	46.2	98.6	96.4	0.001
	Positive	86.1	82.3	58.5	95.3	94.8	
Pap smear–HPV DNA-PCR	Negative	75.0	98.0	66.7	98.6	98.9	0.001
	Positive	94.4	80.0	57.6	98.0	96.1	
HPV DNA-PCR–VIA	Negative	62.5	95.9	45.5	97.9	96.0	0.001
	Positive	86.1	83.2	59.6	95.4	95.6	

VIA test: visual inspection with acetic acid test; HPV DNA-PCR: human papillomavirus deoxyribonucleic polymerase chain reaction; Abnormal histology: ASCUS: atypical squamous cells of unknown significant; CIN2+: cervical intraepithelial neoplasia; and ICC: intraepithelial cervical carcinoma; sensitivity = TP/(TP + FN); specificity = TN/(TN + FP); positive predictive value (PPV) = TP/(TP + FP); negative predictive value (PPV) NPV = TN/(FN + TN), diagnostic accuracy = TP + TN/TP + TN + FP + FN, where TP = true positive, FP = false positive, TN = true negative; FP = false positive and *p* value: probability at the 0.001 level.

## Data Availability

The datasets are available from the corresponding author on reasonable request.

## Additional Points

*Access to Data*. The datasets and questionnaires used in the study can be provided by the corresponding author upon request.
